# Gene Mutation Classification through Text Evidence Facilitating Cancer Tumour Detection

**DOI:** 10.1155/2021/8689873

**Published:** 2021-07-27

**Authors:** Meenu Gupta, Hao Wu, Simrann Arora, Akash Gupta, Gopal Chaudhary, Qiaozhi Hua

**Affiliations:** ^1^Department of Computer Science and Engineering, Chandigarh University, Ajitgarh, Punjab, India; ^2^Digital Zhejiang Technology Operations Co., Ltd., Hangzhou, China; ^3^Bharati Vidyapeeth's College of Engineering, New Delhi, India; ^4^Computer School, Hubei University of Arts and Science, Xiangyang 441000, China

## Abstract

A cancer tumour consists of thousands of genetic mutations. Even after advancement in technology, the task of distinguishing genetic mutations, which act as driver for the growth of tumour with passengers (Neutral Genetic Mutations), is still being done manually. This is a time-consuming process where pathologists interpret every genetic mutation from the clinical evidence manually. These clinical shreds of evidence belong to a total of nine classes, but the criterion of classification is still unknown. The main aim of this research is to propose a multiclass classifier to classify the genetic mutations based on clinical evidence (i.e., the text description of these genetic mutations) using Natural Language Processing (NLP) techniques. The dataset for this research is taken from Kaggle and is provided by the Memorial Sloan Kettering Cancer Center (MSKCC). The world-class researchers and oncologists contribute the dataset. Three text transformation models, namely, CountVectorizer, TfidfVectorizer, and Word2Vec, are utilized for the conversion of text to a matrix of token counts. Three machine learning classification models, namely, Logistic Regression (LR), Random Forest (RF), and XGBoost (XGB), along with the Recurrent Neural Network (RNN) model of deep learning, are applied to the sparse matrix (keywords count representation) of text descriptions. The accuracy score of all the proposed classifiers is evaluated by using the confusion matrix. Finally, the empirical results show that the RNN model of deep learning has performed better than other proposed classifiers with the highest accuracy of 70%.

## 1. Introduction

Gene mutation is defined as the perpetual variation in the normal DNA sequence that is responsible for making up a gene in such a way that the sequence is different from the one that is found in most of the people [1–7]. These gene mutations have variations in sizes, and they can influence every DNA component to a very vast portion of a chromosome that inculcates multiple genes [8]. Some of the genetic disorders caused due to this include cystic fibrosis, colour blindness, and phenylketonuria among multiple others [9]. Cancer has resulted from a sequence of mutations occurring within a single cell. Gene mutations are categorized in two major ways: The first type of mutation is hereditary mutations that are taken from a parent and are there throughout a person's lifespan in virtually every cell present in the body. These are also known as germline mutations as they are available in a parent's germ cells [10]. The other type of mutation is the acquired mutation that forms at some time during the lifetime of a person and is present only in certain cells [11]. These changes are caused when there are some flaws in the DNA copying during cell division or due to certain environmental factors and radiations [12]. Some types of gene mutations are classified as missense, nonsense, insertion, deletion, duplication, and frameshift, among many others. The major effects of a gene mutation include the onset of highly fatal diseases such as cancer [4, 13].

Cancer is caused when the mutation patterns are flawed and becomes malignant for a certain DNA sequence present [14]. The detection of cancer tumours that are formed as a result of gene mutations plays a pivotal role in saving the lives of many people [15, 16]. The gene mutation classification is done manually by the pathologists, but employing an efficient classification model and identifying a gene mutation through textual pieces of evidence would definitely be a breakthrough in mutation classification and subsequently facilitate the detection of cancer tumours.  Figure 1(a) differentiates the structures of normal genes with the mutated genes [17], and Figure 1(b) represents the various levels of genetic mutations [18, 19].

This paper seeks to carry out the classification of the gene mutations through the textual evidence, which would further help in the detection of cancer tumours in an efficient and faster manner as compared to the manual approach followed by pathologists. The text evidence here has been processed by using NLP techniques, which has been a new concept. Further, the application of ML and DL techniques [20, 21] for classification has been incorporated. This work uses three machine learning classification algorithms, Logistic Regression classifier, Random Forest classifier, and Extreme Gradient Boosting (XGB) classifier, along with deep learning Recurrent Neural Network (RNN) classifier [22].

The rest of the paper is organized as follows: Section 2 describes the various researches done in the world related to gene mutations.  Section 3 discusses the exploratory data analysis part, which includes data preprocessing and a detailed data analysis of both the training and the testing datasets.  Section 4 explains the various NLP techniques, text transformation models, and different classification models employed in this research. Various evaluation metrics used, along with a proposed research model, are also discussed in this section.  Section 5 deals with the experimental results and analysis.  Section 6 concludes the entire research and suggests future areas of study.

## 2. Related Work

Cancer is a fatal disease, which, if not detected at the right time, can be extremely painful and cost someone their life. There are countless deaths due to cancer every year worldwide, and the detection in most of the cases is at a crucial stage. It is, therefore, the need of the hour to facilitate the cancer tumour detection methods and save lives. Cancer is caused due to the mutations in genes, which subsequently results in a catastrophic pattern. Several machines and deep learning models are applied and validated to perform the classification of gene mutations efficiently. Some of the researches on the given issue from all over the world are listed in the following.

In [23], Sondka et al. worked on specifying the attributes that would determine the gene present in the Cancer Gene Census (CGC) and its classification regarding these attributes so that their contribution to oncogenesis can be characterized in a better way. In [24], the relationship among the amount of normal stem cell divisions along with the hazard of seventeen types of cancer in sixty-nine countries worldwide was examined.

Further, in [25], Watson and Lynch analysed and reviewed that the male mutation carriers have the colorectal cancer speculation of around 74%. In contrast, the female mutation carriers possess lower speculation, hence having high risk as compared to the general population. Next, in [3], Ali et al. reported that these particular behaviours make the genetic variations in the tumour-suppressing genes, protooncogenes, and oncogenes along with the banal cellular processes handling genes.

Later, in [26], Asano et al. worked on developing the mutant-embellished PCR assay while focusing on exons 19 and 21 of EGFR. In [27], Messiaen et al. studied and performed a test of protein truncation, beginning from puromycin-treated EBV cell lines. They also figured out the germline mutation in sixty-four of sixty-seven patients and the novel thirty-two novel mutations. All the mutations were analysed at the genomic level, as well as the RNA level.

Further, in [28], Forgacs et al. analysed the PTEN|MMAC1, a novel candidate tumour-suppressing gene at 10q23.3, for the mutations in lungs cancer. The PTEN|MMAC1, open reading window of fifty-three lung cancer cell lines, was screened by using the single-stranded conformation polymorphism (SSCP) approach and it was found that it comprised homozygous amino acid sequences that caused the alteration in mutations.

In [29], Coelho, Pinto, and Murray devised a method to emerge genetic uncertainty in the diploid cells of budding yeast *Saccharomyces cerevisiae*, along with isolating the clones with a surge in rates of loss in chromosomes, point mutation, and mitotic recombination. The heterozygous candidate and the mutations causing instability were identified.

Further, in [30], Hollestelle et al. studied and reported a comprehensive molecular characterization of a cluster of forty-one human breast cancer cell lines. Later, in [31], Ma et al. described the correction strategy of heterozygous MYBPC3 (i.e., type of mutation) found in human preimplantation embryos with the specific CRISPR-Cas-stationed accuracy.

After discussing the various researches, this study is focused on the classification of the gene mutations into nine classes, which would further facilitate the detection of cancer tumours through the clinical text evidence provided. Three text transformation models, namely, CountVectorizer, TfidfVectorizer, and Word2Vec, are utilized for the conversion of text to a matrix of token counts. The performance of the proposed framework is determined using the three ML classifiers, namely, LR, RF, and XGBoost, along with the RNN model of DL. This work is in consideration of people's health and to make the detection of gene mutations more efficient than the manual methods [32].

## 3. Dataset Characteristics and Analysis

The dataset for this research work is obtained from Kaggle, which is made available by the Memorial Sloan Kettering Cancer Center (MSKCC) (Kaggle, 2017). Various world-class researchers and oncologists contribute to the preparation of this vast dataset. Two different files are provided in both the training and the testing datasets, among which one file consists of the genetic mutations. In contrast, the other one consists of the clinical evidence (text descriptions) used by the pathologists to classify these genetic mutations into nine classes manually. The attribute ID acts as the connection link between both files. For example, the genetic mutation with corresponding ID = 34 in the file containing genetic mutations has to be classified by using the corresponding entry having ID = 34 in the clinical evidence file [33].

The file containing information about the genetic mutations has four attributes, ID (which acts as the connection link with the clinical evidence file), gene (location of the corresponding genetic mutation), variation (the amino acid change), and 9-label class in which these genetic mutations are classified. Other than this, the file containing the description of clinical evidence has two attributes: one attribute is an ID (which acts as the connection link), and the other one is clinical evidence itself. There are around 3321 samples used for the training purpose, while around 5668 samples are used for the testing purpose. The sample dataset for a file containing information regarding genetic mutation is represented in Table 1.

Both files under the training and the testing datasets are then joined and converted into a single CSV file having five attributes, namely, ID, gene, variation, clinical evidence text, and the class.

The training and testing datasets are checked for the null values, where the total is known, which do not provide any insightful information in the classification task. After the elimination of null values from the training and the testing datasets, we have explored the training dataset for the exploratory analysis of the dataset. The data distribution among the nine classes of the training dataset is shown in Figure 2 which is highly imbalanced. This imbalance situation will be dealt with in this research during the preparation of the classification model by assuring the even split of the training file data into training and testing sets.

The distributions of sentences and words among the nine classes are represented in Figures 3 and 4, respectively.

The comparison of sentence and word distributions among training and testing datasets is shown in Figure 4. In the training set, the peak density is attained in less than 500 sentences per text, whereas, in the testing set, the peak is attained in proximity of the 500 sentences' mark. This shows that the sentence length in the testing set is greater than that in the training set and is achievable in lesser number of sentences. It depicts that, in the training set, the word distribution peak density is attained earlier than in the testing dataset and the density of word length per number of words is less in the training set and comparatively higher in the testing set. However, the difference is not so large and can be avoided.

The training dataset contains 109+153=262 unique genes, while the testing dataset consists of 1243+153=1396 unique genes. Among these, 153 genes are common among the unique genes of both datasets. The counts of the five most mutated genes of all the nine classes are represented in Figure 5.

The training dataset contains 2978+15=2993 unique variations, while the testing dataset consists of 2978+15=5628 unique variations. Among these, 15 variants are common among the unique variation of both datasets. Since the variations in the testing dataset are almost double those in the training dataset, this column is also not very beneficial in the preparation of our classification model. It can be observed that the training dataset contains 436+1596=2032 unique keywords, while the testing dataset consists of 814+1596=2410 unique keywords. Here, 1596 keywords are common among the unique variation of both datasets. It is suggested that the lexical contents of both datasets are almost similar. But it is also observed that some of the keywords, including cells, cell, mutational, mutated, and protein, frequently occur in the dataset but are not so useful for the classification purpose, so there is a need to eliminate them. After the elimination of these unnecessary keywords and other stopwords (which are 433 in total), the dataset contains only the keywords which are useful in the classification purpose.  Figure 6 represents the ten most commonly occurring keywords of all the nine classes in the new dataset, which are free of unnecessary keywords.

## 4. Methodology

In this section, various NLP techniques and three text transformation models, namely, CountVectorizer, TfidfVectorizer, and Word2Vec, along with the various ML and DL classification models, are discussed.

### 4.1. NLP Algorithms and Techniques Employed

Natural Language Processing (NLP) is a technique through which computers understand the natural language that humans use. In NLP, Syntactic Analysis is based on the grammatical aspect of the language and helps to figure out the alignment of natural language with grammatical dogmas [34]. Certain techniques can be used to apply these grammatical rules to the words and infer their meaning [35]. Semantic Analysis is based on the meaning that is conveyed by the text. Understanding the meaning and interpreting the words are done here, along with the structural analysis of sentences [36].

*In CountVectorizer*, the number of times a word occurs in a document is counted [37]. It provides a very lucid way to tokenize the set of text documents along with building a vocabulary of the known words as well as the encoding of fresh documents by making use of that particular vocabulary [38–40]. In *TfidfVectorizer*, the overall weightage of a word occurring in a document is considered [41]. Through this, we can penalize the words that occur most frequently. This is accomplished by taking the product of two metrics, that is, the number of times a word appears in a document and the inverse document frequency of the word across a collection of documents [42]. It uses a measure of how often the words appear in the documents, and the word count is weighted by that measure [43]. It has various use-cases mostly in the scoring of words in the machine learning approaches for Natural Language Processing tasks and the automated analysis of texts. *Word2Vec* (*self-trained and pretrained*) is an algorithm that is used for generating vectors for words [44]. It is a two-layered neural network that is used for processing the text by vectorizing the words [45]. The input provided to it is a corpus of text, and the output produced by it is a collection of vectors, more elaborately, the feature vectors that are the representation of that word in the corpus [46]. Although Word2Vec is particularly not a Deep Neural Network (DNN), it transforms the text into the numerical form that the DNNs can interpret [47].

### 4.2. Classification Model Used

Three machine-learning-based classification models (i.e., LR classifier, RF classifier, and XGB classifier) are used in this research. Parallelly, deep learning classification model, RNN, is also used for the multiclass classification of text (clinical evidence), categorized into nine classes to identify the gene mutation.

#### 4.2.1. Logistic Regression Classifier

It is an ML algorithm that is utilized for categorization problems. This algorithm is based on predictive dissection and the probability concept [2]. The cost function used here is sigmoid rather than a linear function. It limits the cost function between 0 and 1. The sigmoid function (*σ*) and the input (*z*) are determined using the two following equations:

(1) $$\begin{array}{c} \sigma \left(x\right)=\frac{1}{1+e^{-z}}, \end{array}$$

(2) $$\begin{array}{c} z=w_{0}x_{0}+w_{1}x_{1}+\cdots +\;w_{n}x_{n}+\text{bias,} \end{array}$$

where *z* is the resultant number obtained by the multiplication of *x*, which is the input vector provided, and *w*, which represents the coefficients along with the addition of a bias factor.

#### 4.2.2. Random Forest Classifier

RF is a classification algorithm that consists of several decision trees. When constructing, each particular tree in the forest makes a class prescience, and the class with the maximum votes becomes the prediction of our model [5]. It uses bagging and features randomness to try to establish an uncorrelated forest of trees whose forecast by committee is more reliable than that of any single tree [48].

#### 4.2.3. XGB Classifier

Extreme Gradient Boosting, also known as XGBoost, is an ensemble machine learning algorithm that is based on decision trees [49]. It utilizes a gradient boosting approach. Gradient boosting is a method where new models are generated to calculate the residuals or errors of previous models and then summed up to produce the final prediction [50]. This is known as gradient boosting, since it uses an algorithm of gradient descent to reduce the loss while introducing new models.

#### 4.2.4. RNN Classifier

RNN is defined as the artificial neural network which can be interpreted as a sequence comprising blocks of neural networks linked to each other in a chain manner [51]. This particular architecture facilitates RNN to show temporal behaviour and sequentially captivate the data, which is a more acceptable approach in text classification as the text is mostly in a sequential form [1].

### 4.3. Proposed Methodology

Figure 7 represents the proposed model of our research work. Initially, both the training and the testing datasets provided by the Kaggle team are checked for the null values and are analysed in detail. After the completion of data cleaning and analysis, three text transformation models, namely, CountVectorizer, TfidfVectorizer, and Word2Vec, are utilized for the conversion of text to a matrix of token counts. Three ML classification models, namely, LR, RF, and XGBoost, along with the RNN model of DL, will then be applied to the sparse matrix (keywords count representation) of text descriptions. The training file is evenly split into training and testing sets. It is split in the way such that the test set also contains the examples of all the 9 classes. Then, all the proposed classifiers are empirically compared by determining the accuracy score with the help of the confusion matrices [52] and accuracy scores [53]. Finally, the classifier model with the highest accuracy score is determined.

## 5. Experimental Results and Analysis

In this section, three text transformation models, namely, CountVectorizer, TfidfVectorizer, and Word2Vec, are utilized for the conversion of text to a matrix of token counts.

### 5.1. Machine Learning Classifiers

Three machine learning classifiers, namely, Logistic Regression, Random Forest, and XGBoost, are applied to the sparse matrix of clinical evidence text [54].

#### 5.1.1. CountVectorizer

CountVectorizer class from the feature_extraction.text module of the sklearn library is used for the conversion of clinical evidence text to a series of token counts. It uses CountVectorizer class to count the occurrence of each word. All three proposed machine learning classifiers are then trained and compared by using the accuracy score obtained by the confusion matrix [55]. The total number of features in this text transformation model is calculated to be 157815.

*(1) Logistic Regression*. In the Logistic Regression algorithm, initially, the features are standardized by using the StandardScalar class from the sklearn library. After that, the count vectors obtained from the sparse matrix are fitted to the Logistic Regression model, and the test scores are calculated by tuning parameter *c*, which is defined as the inverse of the regularization strength [56–61]. The best value of *c* comes out to be 0.001, at which the model shows its optimum performance.  Figure 8 represents the average accuracy score and confusion matrix of the proposed Logistic Regression classifier, along with the individual accuracy scores of all the nine classes. The average accuracy score for this model is coming out to be 38.15%.

*(2) Random Forest*. In the Random Forest classification algorithm, the count vectors obtained from the sparse matrix are fitted, and the test scores are calculated by tuning the various parameters to achieve the optimum performance of the model. The optimum values of parameters are as follows: n_estimators (total number of trees used) = 1000, max_depth (maximum depth of the tree) = 20, and min_samples_leaf (minimum number of required samples at a leaf node) = 5.  Figure 9 represents the average accuracy score of the proposed Random Forest classifier, along with the individual accuracy scores of all the nine classes. The average accuracy score for this model is coming out to be 47.47%.

The confusion matrix of the Random Forest classifier for the CountVectorizer text transformation model is shown in Figure 10.

*(3) XGB Classifier*. In the XGBoost classification algorithm [62–66], the count vectors obtained from the sparse matrix are fitted, and the test scores are calculated by tuning the various parameters to achieve the optimum performance of the model. The optimum values of the various parameters are as follows: eta (learning rate) = 0.05, minimum loss reduction = 0.4, max_depth (maximum depth of the tree) = 6, min_child_weight (minimum sum of instance weights in a child) = 10, and colsample_bytree (the subsample ratio) = 0.6.

The average accuracy score and confusion matrix of the XGBoost classifier for the CountVectorizer text transformation model are shown in Figure 11. This model shows the highest accuracy score of 48.49% among all the machine learning models for the CountVectorizer text transformation model.

#### 5.1.2. TfidfVectorizer

TFIDF stands for term frequency-inverse document frequency. TfidfVectorizer class from the feature_extraction.text module of the sklearn library is used for the conversion of clinical evidence text to a series of token counts. TFIDF can normalize the word count in any document against the total number of documents containing that word in the entire corpus. All three proposed machine learning classifiers are then trained and compared by using the accuracy score obtained by the confusion matrix. The total number of features in this text transformation model is calculated to be 157815.

*(1) Logistic Regression*. In the Logistic Regression algorithm, initially, the features are standardized by using the StandardScalar class from the sklearn library. After that, the count vectors obtained from the sparse matrix are fitted to the Logistic Regression model, and the test scores are calculated by tuning parameter *c*, which is defined as the inverse of the regularization strength. The best value of *c* comes out to be 0.001, at which the model shows its optimum performance.

Figure 12 represents the average accuracy score and confusion matrix of the proposed Logistic Regression classifier, along with the individual accuracy scores of all the nine classes. The average accuracy score for this model is coming out to be 38.54%.

*(2) Random Forest*. In the Random Forest classification algorithm, the count vectors obtained from the sparse matrix are fitted, and the test scores are calculated by tuning the various parameters to achieve the optimum performance of the model. The optimum values of the various parameters are as follows: *n*_estimators = 500, max_depth = 20, and min_samples_leaf = 1.  Figure 13 represents the average accuracy score and confusion matrix of the proposed Random Forest classifier, along with the individual accuracy scores of all the nine classes. The average accuracy score for this model is coming out to be 48.28%.

*(3) XGBoost*. In the XGBoost classification algorithm, the count vectors obtained from the sparse matrix are fitted, and the test scores are calculated by tuning the various parameters to achieve the optimum performance of the model. The optimum values of the various parameters are as follows: eta (learning rate) comes out to be 0.05, gamma = 0.4, max_depth = 6, min_child_weight = 5, and colsample_bytree = 0.2.

Figure 14 represents the average accuracy score and confusion matrix of the proposed XGBoost classifier, along with the individual accuracy scores of all the nine classes. This model shows the highest accuracy score of 49.73% among all the machine learning models for the TfidfVectorizer text transformation model.

#### 5.1.3. Word2Vec

In this section, the Word2Vec text transformation model is used for the training of the embedding matrix. As the name suggests, in this model, initially, each word is represented by a numeric vector. The embedding size is taken as 100; that is, each word is represented by the numeric vector of 100 dimensions. After that, all the numeric vectors are averaged to get a single vector for each of the documents. In this research, we use gensim.models.Word2Vec for the training purpose. All three proposed machine learning classifiers are then trained and compared by using the accuracy score obtained by the confusion matrix.

*(1) Logistic Regression*. In the Logistic Regression algorithm, initially, the features are standardized by using the StandardScalar class from the sklearn library. After that, the count vectors obtained from the sparse matrix are fitted to the Logistic Regression model, and the test scores are calculated by tuning parameter *c*, which is defined as the inverse of the regularization strength. The best value of *c* comes out to be 0.01, at which the model shows its optimum performance.

Figure 15 represents the average accuracy score and confusion matrix of the proposed Logistic Regression classifier, along with the individual accuracy scores of all the nine classes. The average accuracy score for this model is coming out to be 46.71%.

*(2) Random Forest*. In the Random Forest classification algorithm, the count vectors obtained from the sparse matrix are fitted, and the test scores are calculated by tuning the various parameters to achieve the optimum performance of the model. The optimum values of the various parameters are as follows: max_depth = 5 and min_samples_leaf = 5.

Figure 16 represents the average accuracy score and confusion matrix of the proposed Random Forest classifier, along with the individual accuracy scores of all the nine classes. The average accuracy score for this model is coming out to be 45.02%.

*(3) XGBoost*. In the XGBoost classification algorithm, the count vectors obtained from the sparse matrix are fitted, and the test scores are calculated by tuning the various parameters to achieve the optimum performance of the model. The optimum values of the various parameters are as follows: min_child_weight = 5 and colsample_bytree = 1.

Figure 17 represents the average accuracy score and confusion matrix of the proposed XGBoost classifier, along with the individual accuracy scores of all the nine classes. This model shows the highest accuracy score of 48.22% among all the machine learning models for the Word2Vec text transformation model.

### 5.2. Deep Learning Classifiers

Along with three machine learning models, the RNN model of deep learning is also applied to the sparse matrix of clinical evidence text.

#### 5.2.1. RNN Model with Pretrained Word2Vec

In this method, pretrained word vectors are used for the conversion of each word to a numeric vector. The visualization of the training performance can be seen in Figure 18. It can be observed from Figure 18 that even though the training loss has been reduced, the validation loss has been improved. Also, it shows that the validation accuracy is lower than that of the training accuracy.

Figure 10 represents the average accuracy score and confusion matrix of the proposed RNN classifier with pretrained Word2Vec, along with the individual accuracy scores of all the nine classes. This model shows the highest accuracy score of 70.78% among all the proposed models in this research.

#### 5.2.2. RNN Model with Self-Trained Word2Vec

In this method, instead of using pretrained vectors, the Word2Vec transformation model is trained using the available dataset. After that, the RNN model is trained, and its performance is evaluated by using the confusion matrix. The visualization of the training performance can be seen in Figure 19. It can be observed from Figure 19 that even though the training loss has been reduced, the validation loss has been improved. Also, it shows that the validation accuracy is lower than that of the training accuracy.

The accuracy scores and confusion matrix of the RNN classifier with a self-trained Word2Vec text transformation model are shown in Figure 20. The average accuracy score for this model is 67.77%, which is a little bit less than that with the pretrained Word2Vec but high as compared to the machine learning models.

## 6. Conclusion and Future Enhancement

This research work is carried out to propose a multiclass classifier to classify the genetic mutations based on the clinical evidence, that is, the text description of these genetic mutations, which helps in the distinguishing of drivers with passenger genetic mutations. It also helps out in the development of personalized medicine for cancer treatment. NLP techniques are employed in this research to build this multilabel classifier. Three text transformation models, namely, CountVectorizer, TfidfVectorizer, and Word2Vec, are utilized for the conversion of text to a matrix of token counts. The performance of the proposed framework is determined using the three machine learning classification models, namely, LR classifier, RF classifier, and XGB classifier, along with the RNN model of deep learning. The performance is evaluated using the confusion matrix. Finally, the empirical results show that the RNN model of deep learning with a pretrained Word2Vec text transformation model performed better than the other proposed classifiers with the highest accuracy of 71%. The model would possibly lead to the detection of cancer tumours in an efficient and faster manner as compared to the manual approach followed by pathologists.

The proposed model can be enhanced in the future by incorporating the other text transformation models like truncated singular value decomposition (SVD) and Doc2Vec for the text conversion. Along with this, other machine learning classifiers like Multinomial Naïve Bayes, Support Vector Machine, and Deep Learning classifiers (LSTM, Conv1D, and Gated Recurrent Units) can be applied to the sparse matrix which can lead to an increase in the model efficiency.

## Figures and Tables

**Figure 1:** (a) Comparison of normal and mutated genes [17]. (b) Different levels of genetic mutations [18].

**Figure 2:** Distribution of the training file data among the nine classes.

**Figure 3:** (a) Total number of sentences in the nine classes. (b) Total number of words in the nine classes.

**Figure 4:** Comparison of training and testing datasets. (a) Sentences distribution and (b) words distribution.

**Figure 5:** The counts of the five most mutated genes of all the 9 classes.

**Figure 6:** Ten most commonly occurring keywords of all the nine classes.

**Figure 7:** Flow of proposed methodology.

**Figure 8:** Logistic Regression classifier for the CountVectorizer text transformation model. (a) Accuracy scores. (b) Confusion matrix.

**Figure 9:** Random Forest classifier for the CountVectorizer text transformation model. (a) Accuracy scores. (b) Confusion matrix.

**Figure 10:** RNN classifier with a pretrained Word2Vec text transformation model. (a) Accuracy score. (b) Confusion matrix.

**Figure 11:** XGBoost classifier for the CountVectorizer text transformation model. (a) Accuracy scores. (b) Confusion matrix.

**Figure 12:** Logistic Regression classifier for the TfidfVectorizer text transformation model. (a) Accuracy scores. (b) Confusion matrix.

**Figure 13:** Random Forest classifier for the TfidfVectorizer text transformation model. (a) Accuracy scores. (b) Confusion matrix.

**Figure 14:** XGBoost classifier for the TfidfVectorizer text transformation model. (a) Accuracy scores. (b) Confusion matrix.

**Figure 15:** Logistic Regression classifier for the Word2Vec text transformation model. (a) Accuracy scores. (b) Confusion matrix.

**Figure 16:** Random Forest classifier for the Word2Vec text transformation model. (a) Accuracy scores. (b) Confusion matrix.

**Figure 17:** XGBoost classifier for the Word2Vec text transformation model. (a) Accuracy scores. (b) Confusion matrix.

**Figure 18:** Training and validation loss for RNN model with pretrained Word2Vec. (a) Loss plot. (b) Accuracy.

**Figure 19:** Training and validation for RNN model with self-trained Word2Vec. (a) Loss plot. (b) Accuracy.

**Figure 20:** RNN classifier with a self-trained Word2Vec text transformation model. (a) Accuracy scores. (b) Confusion matrix.

**Table 1:** Sample dataset for the file containing a description of genetic mutations.

ID	Gene	Variation	Class
0	FAM58A	Truncating mutations	1
1	CBL	W802	2
2	CBL	Q249E	2
3	CBL	N454D	3
4	CBL	L399V	4
5	CBL	V391I	4
6	CBL	V430M	5
7	CBL	Deletion	1
8	CBL	Y371H	4

## Data Availability

The dataset for this research work is obtained from Kaggle, which is made available by MSKCC. Data are available at https://www.kaggle.com/c/msk-redefining-cancer-treatment/data.
